The article "Research on the New Ecological Model under the Environment of “Double Reduction” of Children's Community Education Services" was published in 2022. Journal: J Environ Public Health.

# Research on the New Ecological Model under the Environment of “Double Reduction” of Children's Community Education Services

**DOI:** 10.1155/2022/9471160

**Published:** 2022-07-08

**Authors:** Jing Zhou

**Affiliations:** School of Humanities, Geely University of China, Chengdu 641402, Sichuan, China

## Abstract

Children are the hope of building a powerful, modern-socialist state. In recent years, all social classes have paid more and more attention to children's enlightenment education, and the country began to implement the double reduction policy. As the main place for children to live and grow, the community has the responsibility and obligation to conduct the education of children. Work and effective development and utilization of community education resources can greatly meet the needs of children's growth, help children develop good behavior habits, and lay a solid foundation for future education. Through the experimental survey results, this paper discusses the theoretical basis for the development and utilization of community children's education resources under the dual emission reduction policy, puts forward the corresponding development principles, and analyzes the main strategies to improve the efficiency of social education.

## 1. Introduction

In recent years, in accordance with the decisions and arrangements of the Party Central Committee and the State Council, all localities have carried out in-depth efforts to reduce the burden of homework and off-campus training (hereinafter referred to as “double reduction”) for students in the compulsory education stage [1]. But one of the most prominent problems in compulsory education now is that primary and secondary school students are too burdened, and the problems of short-sightedness and utilitarianism have not been fundamentally resolved [2]. On the one hand, students' homework burden is still heavy, and homework management is not perfect; on the other hand, off-campus training is still overheated, and the problem of advanced and overstandard training has not been fundamentally resolved [3]. Illegal behaviors, such as “difficulty in refunding fees” and “running away with money” by training institutions, have occurred from time to time [4]. These problems have resulted in the heavy burden of students' homework and off-campus training and the heavy financial and energy burden of parents, which has seriously offset the achievements of educational reform and development, and it has had a very bad impact on society [5]. The Party Central Committee attaches great importance to this, and from the strategic height of realizing the great rejuvenation of the Chinese nation, it has made important decisions and arrangements for the “double reduction” work. Education policy implements the fundamental task of Lide Shuren and promotes the all-round development and healthy growth of students [6]. At present, my country's educational undertakings have been vigorously developed [7]. The Party Central Committee has paid more and more attention to children's education, actively developed and utilized community educational resources, improved the community's ability to guide children's education, and strived to create a learning, friendly, and united community [8]. Educational atmosphere: However, in the process of developing and utilizing community educational resources, there are also problems such as unclear goals, difficulty in developing resources, and uncooperative personnel [9]. Therefore, it is necessary for the community to strengthen management, clearly recognize the importance of community educational resources to children's growth, and actively develop and use effective community education resources to create a good environment for children's growth and learning [10].

The article "Research on the New Ecological Model under the Environment of “Double Reduction” of Children's Community Education Services" was published in 2022. Journal: J Environ Public Health.

Parents and students get along day and night. As the children's second teachers, their words and deeds also affect the children's learning [11]. It is very important to fulfill their legal guardianship duties. First, open home-school contact [12]. Actively participate in parent meetings and parent schools, actively communicate with teachers, understand students' learning and physical and mental conditions, formulate targeted home-school linkage education programs, and build a harmonious home-school relationship [13]. The second is to update the concept of parenting. Understand the law of children's physical and mental growth, improve their own educational quality and ability, rationally plan the future development direction of children, and do not blindly send children to participate in off-campus training [14]. The third is a harmonious family atmosphere. Carefully pay attention to the changes in children's thoughts and emotions, listen to their voices, be their friends, form a good communication and interaction model, and help children solve problems [15]. The fourth is to guide students to make good use of their time at home. Encourage your child to go to bed on time and ensure adequate sleep [16]. Moderately arrange housework, strengthen physical exercise, carry out parent-child reading, etc. Strengthen the supervision of children's online behavior and timely detect, stop and correct children's online addiction [17].

Society is the environment of education, and it is necessary to give full play to the resources of all parties to provide an important platform for students to broaden their horizons, develop in an all-around way, and practice exercises [18], as shown in Table 1.

The article "Research on the New Ecological Model under the Environment of “Double Reduction” of Children's Community Education Services" was published in 2022. Journal: J Environ Public Health.

## 2. Relevant Theoretical Basis for the Development and Utilization of Community Educational Resources

The development and utilization of community education resources are not blind but also need to be guided by a relevant theoretical basis.  Figure 1 contains three aspects: ecological theory, constructivism theory, and the theory of “life education.”

### 2.1. Ecological Theory

Bronfenbrenner, the founder of human development ecology, believes that “The environment in which individuals develop is an ecosystem that spreads from small to large, and each system affects the development of individuals in a certain way. These environments exist specifically in the life of individual development in different forms, such as schools, families, communities, the entire social culture, and the interaction process and connection between individuals and their environment and between environments and environments [19]. This theory reveals to us that schools, families, and communities all have important influences on children's development. Long recognized and valued for the vital role of the family and school for children, now we need to recognize the important influence of communities in children's development. The lives and development of children are influenced by the community, and this influence becomes more widespread as the child matures. The magnitude of this influence also depends on how the community develops and utilizes various resources [20].

The ecosystem is the place where human beings live and grow. Human life is a group, and it is difficult for any individual to grow and develop without society and others. In the theory of human development ecology, it is proposed that the development environment of each person is a system that expands layer by layer from small to large, and each layer of the system will have a certain impact on the growth and development of the individual. These influences include families, schools, communities, etc., and the systems at all levels also interact to bring learning and living resources to individual growth. From the ecological theory, it can be seen that the community plays an important role in the growth stage of children, which will have a great impact on children's thinking, cognition, and behavior habits. More extensive and far-reaching, this impact will also depend on the development and utilization of community educational resources. The effective development and utilization of educational resources will guide children to establish correct thinking and cognition and play a positive role; otherwise, it will be detrimental to children.

The article "Research on the New Ecological Model under the Environment of “Double Reduction” of Children's Community Education Services" was published in 2022. Journal: J Environ Public Health.

### 2.2. The Theory of Constructivism

Constructivism is a theory about knowledge and learning, which emphasizes the initiative of learners, and believes that learning is a process in which learners generate meaning and construct understanding based on the original knowledge and experience. The constructivist theory originates from the study of cognitive development and has important implications for understanding the process of children's learning and development. The two representatives of constructivism are Piaget and Vygotsky. Piaget emphasized individual construction and believed that the development of children's cognition stemmed from the interaction of subject and object. He emphasized that “the action of the subject, that is, the interaction between the subject and the object, is the source of all experience and knowledge. Only when children act on the environment can the development of their cognitive structure be guaranteed.” Piaget advocated that children learn through active manipulation of physical objects, Encouraging children to discover problems by themselves, formulate their own hypotheses, collect data and verify their own conclusions, and provide children with a rich and diverse educational environment. These ideas can be a guide for child caregivers. Vygotsky emphasizes social construction and believes that social culture has an important influence on children's knowledge construction. “Vygotsky believed that the establishment of all higher cognitive processes results from mutual contact with society. By participating in the common activities of more mature members of society, children gradually master these activities and develop them in ways that are meaningful in their culture. Way of thinking.” Piaget and Vygotsky emphasized that children's development is achieved through the manipulation of things and interaction with people, so in the process of developing and utilizing community educational resources, educators need to actively develop and utilize things and the elements of people.

Constructivism theory mainly originates from the study of human cognition and plays an important guiding role in the development and utilization of children's educational resources. This theory holds that the development of children's cognition is mainly affected by the interaction between the subject and the object. When children act in the living environment, their cognitive construction will be greatly improved. At the same time, the development of children's cognition is a process of continuous exploration and creation. Children need to operate in the living environment, discover problems, put forward hypotheses, explore problems, and finally draw conclusions, or solve problems. Therefore, the community can provide enough knowledge answers for children by establishing a community children's library, interest corner, and other ways— a place that satisfies children's exploration and cognition of the world. In addition, Vygotsky, a researcher of constructivism theory, believes that social culture also plays an important role in children's growth and cognitive construction and proposes that all more advanced cognitive processes need to be in contact with society. Only when members communicate with each other can they help children deeply understand social life and culture.

The article "Research on the New Ecological Model under the Environment of “Double Reduction” of Children's Community Education Services" was published in 2022. Journal: J Environ Public Health.

### 2.3. The Theory of “Living Education.”

The life educational theory system is composed of the purpose, principle, and basic way of life education, as shown in Figure 2. Mr. Chen Heqin, a Chinese children's educator, studied a series of excellent foreign educational theories and ideas while studying in the United States. After returning to China, he devoted himself to Sinicization and scientific exploration of advanced educational ideas and put forward the theory of “living education” according to China's national conditions. In the theory of “living education,” Chen Heqin emphasizes that “nature and society are living textbooks.” Chen Heqin believes that knowledge in books is indirect and formalized, and only nature and society are the real sources of knowledge. A living book, a living textbook. Chen Heqin uses nature and society as teaching materials for living education, as shown in Table 2. On the one hand, because nature and society are the sources of knowledge, the knowledge it provides to children is the most vivid, intuitive, and vivid, and it avoids any formalized links and artificial intelligence. It is easy to form children's correct concept of things. On the other hand, education that fits children's life through nature and society is also the education that can stimulate children's interests the most. Children like to be active in nature and the big society. Nature and society are the worlds of children and the environment in which children live. In view of the importance of nature and society in the development of children, we should pay full attention to these two factors in the development and utilization of social educational resources.

Therefore, the development and utilization of community educational resources are of positive significance to children's growth and life. It has strong theoretical support and has been explored and researched by countless people, which is in line with the psychological characteristics and interests of children's learning.

## 3. Principles of Development and Utilization of Educational Resources for Children in the Community

Some principles also need to be upheld in the development and utilization of community children's educational resources, as shown in Figure 3, including the following three principles, which will be introduced later.

The article "Research on the New Ecological Model under the Environment of “Double Reduction” of Children's Community Education Services" was published in 2022. Journal: J Environ Public Health.

### 3.1. The Principle of Subjectivity

The so-called principle of subjectivity means that children should be the main body in the development and utilization of community educational resources, breaking the previous state of being dominated by adults, and must fully consider the characteristics and needs of children. Dewey once pointed out that children have four instincts, namely, the instinct of inquiry, the instinct of social interaction, the instinct of art, and the instinct of manufacture. The positive growth of children depends on the realization of these instincts. In these instinctive activities, children's interests are stimulated, and their subjectivity is fully exerted. The inspiration from Dewey's point of view is that in the development and utilization of community educational resources, we should take into account the realization of children's instincts and arrange objects for inquiry, social space, artistic atmosphere, and production opportunities.

In the past, the community education method was relatively backward, and the teaching mode was relatively simple and outdated. Some communities did not fully develop and utilize educational resources and did not pay attention to children's teaching, making it difficult for children to play their dominant position; children lose the initiative to learn, have no interest in community teaching, and overtime will also produce boredom, which is not conducive to children's growth and learning. Therefore, the development and utilization of community educational resources need to adhere to the principle of children as the main body, clarify the main position of children in the development and utilization of community educational resources, take children as the core, and explore and utilize educational resources from the perspective of children. Break through the stereotyped or adult-led education model. Children have the instincts of inquiry, socialization, art, and manufacture. Therefore, the community needs to provide more facilities and equipment for children so that children can explore and learn independently. For example, place exploration materials, or facilities in the square so that children can make the desired item.

### 3.2. The Principle of Suitability

The so-called suitability principle refers to the suitability of community educational resources for children. This suitability includes two aspects: one is the suitability of the age, and the other is the suitability of the individual, as shown in Figure 4.

The article "Research on the New Ecological Model under the Environment of “Double Reduction” of Children's Community Education Services" was published in 2022. Journal: J Environ Public Health.

Age suitability emphasizes that the community should have educational resources for children of different ages, such as suitable venues and pavements for toddlers and safe large sports venues and facilities for children aged 2–6.

Individual suitability emphasizes that community resources should consider different individual needs. There are various types of resources that can meet the individual needs of children. For example, sports resources meet the needs of sports children, library resources meet the needs of reading children, and science and technology museum resources meet the needs of exploratory children.

The development and utilization of community educational resources must be suitable for children's growth and development, and scientific and reasonable teaching materials should be provided according to children's psychological characteristics and interests. First of all, the community should start from the age of the children. Generally speaking, the general age of children is between one and six years old. They are curious, eager to learn, and have a strong interest in learning new things. Therefore, the development of community education resources should be divided into different types according to the age group of children. For example, children aged 1–4 should teach them to know things, give them innovation and freshness, provide surprises at any time, and stimulate their enthusiasm for learning. Secondly, children's education should not be rushed, it should be done gradually, and it is too late. According to the needs of children's age, they should be provided with suitable teaching resources. At the same time, the infrastructure should also meet the learning needs of children. The development and utilization of community resources cannot rely solely on adults. Willingness should fully consider the growing needs of children and provide fresh and suitable learning resources in order to guide children to grow up healthily in the community.

### 3.3. The Principle of Development

The so-called developmental principle refers to meeting the actual needs of children while focusing on the future development of children. The development and utilization of community resources do not only focus on the visible transient development of children but also on the sustainable development of children. At the same time, the developmental principle is also reflected in promoting the overall development of children rather than one-sided development. For a long time in the past, adults have paid much attention to the cognitive development of children and neglected the development of emotions and skills. Holistic development requires attention to the harmonious development of children's cognition, emotion, and skills. According to Gardner's theory of multiple intelligences, every child has multiple intelligences, but each child exhibits different dominant bits of intelligence. In order to meet the group needs of children's development, the community needs to have rich and diverse resources and to meet the individual needs of children's development. The community needs to have individualized resources and community organizations, to answer questions about children's personal development at different stages or to provide some effective advice on their personal development according to their own interests. The diversification and individualization of community educational resources will promote the individualized development of children.

The article "Research on the New Ecological Model under the Environment of “Double Reduction” of Children's Community Education Services" was published in 2022. Journal: J Environ Public Health.

The development and utilization of community educational resources need to focus on the future development and growth of children. It cannot provide children with flashy educational resources. It should proceed from reality and keep pace with the times, keep up with the trend of the times, and combine the most cutting-edge and cutting-edge educational resources. Advanced concepts of children's education uphold the principle of child development so as to ensure the continuity and long-term nature of community education resources. The development and utilization of community educational resources should be based on the overall situation, not just the current and one-sided attention. In the past development of community educational resources, some communities ignored the developmental principle, and the learning resources provided for children lacked integrity. At the same time, they paid too much attention to children's cognitive and behavioral abilities and often neglected to cultivate children's emotions. Therefore, the community needs to provide children with a variety of learning resources according to the needs of children's development, cultivate and improve children's behavior habits and emotional cognition, and ensure the development and utilization of community educational resources. Diversified and personalized enrichment development.

## 4. Strategies for the Development and Utilization of Educational Resources for Children in the Community

According to the relevant theory and principle analysis mentioned above, the strategies shown in Figure 5 can be used in the development and utilization of community educational resources for children.

### 4.1. Development and Utilization of Natural Resources

Every community is different, but all have certain natural resources. Natural resources generally refer to the natural conditions (natural environment elements) that exist in nature and can be used by human beings, including land resources, water resources, climate resources, and biological resources. There are three main reasons for the development of resource resources.

The article "Research on the New Ecological Model under the Environment of “Double Reduction” of Children's Community Education Services" was published in 2022. Journal: J Environ Public Health.

#### 4.1.1. Natural Resources Provide Children with Rich Emotional Experiences

Children may live in cities, suburbs, or rural areas, and each type of community has different resources, but all provide a rich emotional stimulus for child development, and children can observe different aspects of nature in their own communities. Children in rural areas can see small animals, such as poultry, livestock, and various types of crops, and they can also see cute insects such as butterflies, bees, and dragonflies more easily; children in cities can see many open parks. Flowers in the garden and animals in the zoo, etc. Children in the north see poplar, willow, and locust trees more often; children in the south see plane trees, camphor trees, and osmanthus trees more often. The natural climate also provides learning materials. Children living in coastal areas are more likely to experience typhoons, and children living inland are more likely to feel the pain of drought. In the community, children can directly experience the feelings brought by the change of the four seasons of natural objects, including the vitality of all things in spring, the colorful flowers in summer, the fragrance of sweet-scented osmanthus and ginkgo leaves in autumn, and the cold wind and rain in winter. Snow is flying.

#### 4.1.2. Natural Resources Provide a Source of Mental Development for Children

The Soviet educator Suhomlinsky pointed out affectionately: If children want to get training in thinking, they have to travel to nature. In nature, children's minds become active, and they perceive both the obvious interconnections between phenomena in the world around them, as well as those that are not immediately apparent. Gradually, this initial concept of living and nonliving things is formed in the child's consciousness. Some things are living things, and other things are nonliving things - this is something children can see through a lot of facts. In the process, things in nature become the source of children's thinking development. Children see and experience nature with their own eyes, constantly pay attention to and think about natural objects, and explore causal connections, and the original concrete visualization thinking gradually develops into abstract logical thinking. All-natural objects in the community can become a stream of distinct objects, perceptions, and representations flowing into the hearts of children's thinking, thus forming a certain impact on the children's mental health.

The article "Research on the New Ecological Model under the Environment of “Double Reduction” of Children's Community Education Services" was published in 2022. Journal: J Environ Public Health.

### 4.2. Development and Utilization of Space Resources

The community is an important place in children's life. Each community contains basic venues and various institutional facilities. These spaces can also be constructed as children's learning fields.

#### 4.2.1. Community Public Spaces Provide Opportunities for Children to Exercise and Communicate

Public spaces are standard in every community, but there are large and small differences. With the development, a lot of space is occupied by private people, and there is less and less public space. Sometimes someone takes the space privately because it is also money, and sometimes it is a fringe, no identity, full of parked vehicles, trash cans, or signage. The way spaces were used in the past had to be changed and given quality and value to them. A good community should have public spaces where children can move freely. Public spaces need to be safe, spacious, open, and accessible. Many separate areas can be set up in the public area to meet children's sports interests, such as a water play area, sand play area, sports area, and equipment for children's sports can also be added in the corresponding areas. Children play to their heart's content in public areas to achieve full physical movement. At the same time, children get to know a wide range of members of the community in public places and gain social development through communication with them.

#### 4.2.2. Public Service Agencies in the Community Provide Opportunities for Children's Social Cognition

These public service agencies provide services to each family and provide children with opportunities for social awareness through formal and informal means, as shown in Table 3. These institutions serve as educational bases for children and can arrange specialized staff to give professional demonstrations and guidance to children. Studies have shown that children who are able to go to zoos, parks, museums, libraries, and corporate buildings perform better in various school subjects than children who do not have the opportunity. In these public service institutions, children also gain specific perceptions of the social roles and behaviors of institutional staff, laying an empirical foundation for them to understand and adapt to society. For example, the police can educate children about safety and guide them to protect themselves; police can put on uniforms to show their working status and tools, teach children how to contact the police in time when they are in danger, and teach children how to cooperate when police help is needed. When children go shopping in the supermarket, children can gain rich mathematical experience, including specific experiences, such as item type, quantity, size, production date, etc.

The article "Research on the New Ecological Model under the Environment of “Double Reduction” of Children's Community Education Services" was published in 2022. Journal: J Environ Public Health.

### 4.3. Development and Utilization of Human Resources

According to the point of view of symbolic interaction theory, the interaction between people is based on the interaction of symbols, and the symbol is the mediator of the interaction. Human behavior is meaningful, and to understand a behavior, we must make a concrete explanation of the meaning that the actor assigns to his behavior. The inspiration given to us by this point of view is that we should pay full attention to the mediating role of symbols, use symbols appropriately, and at the same time listen to the interpretation of the symbols by the behavior sender and understand the meaning of the other party's behavior. All of this needs to be realized in interaction. Children understand the value and meaning of symbols in their interaction with others and enhance their own social experience.

#### 4.3.1. Children Gain Social Experience in Their Interactions with Adults

Children's interactions with adults in the community affect children's development because children learn a range of different social patterns and gain different experiences in the process of interacting with adults.

*(1) Professional Educators Provide Professional Education Guidance*. Every community has various types of educational institutions, and teachers in educational institutions are professional educators. They can play a more active role in educating children. On the one hand, professional educators can provide advice and suggestions for community children's education; on the other hand, professional educators can provide educational services for community children in their spare time. Professional educators can provide advice to parents, solve troubles for children, and organize rich activities for children to build a platform for children to grow. Professional educators' community service can be incorporated into their work performance, gaining practical experience in education and recognition at work. Professional educators actively participate in community children's education, which will promote the common growth of children, parents, and professional educators themselves. For example, the Sihuan Game Team, founded by graduate students of Beijing Normal University in a vegetable market in Beijing, has achieved good social and professional growth effects.

*(2) People in Various Industries Provide Vocational and Labor Education*. Community people are widely distributed in all walks of life, and the work experience of people from all walks of life can be a source of learning for children in the community. People from all walks of life have their own expertise, and they can use their expertise to contribute to the education of children in the community. For example, doctors can educate and guide children in the common sense of medical and healthcare; lawyers can publicize children's knowledge of the law, abide by the law, understand the law, and use it; sports workers can form sports teams to lead children in professional sports, etc. The community can recruit volunteers to mobilize the power of people from all walks of life and form various learning and sports groups to promote children's development. In contact with people in various industries, children learn about relevant occupational roles and behaviors and carry out observational learning. The daily operation of life requires the labor of people from all walks of life to maintain. Children in all walks of life can directly feel the importance and glory of labor and then gradually develop a love for labor and respect for the fruits of labor. Children gain a perceptual understanding of occupations from their interactions with people in various industries, gradually clarify their career choices, and lay a preliminary experience for future development and employment.

The article "Research on the New Ecological Model under the Environment of “Double Reduction” of Children's Community Education Services" was published in 2022. Journal: J Environ Public Health.

#### 4.3.2. Children Develop Social Behaviors in Interactions with Peers

Children are naturally gregarious, and they cannot grow without interaction with their peers. Peer groups will provide children with early experiences of social interaction and cooperation and promote their social development. In the case of limited resources, children and peers will compete, such as competing for venues, equipment, and partners. But more often, there is a cooperative relationship between children and their peers. They cooperate in games and sports, learn to adapt to each other under the rules of turns and exchanges and gain social interaction experience. There is an equal dialogue relationship between children and their peers. They support each other, help each other, learn from each other, share experiences and troubles, and achieve common growth. Friends are very important to every child in his childhood. When children become adults, they still cherish the friendship of their childhood peers, which has become a good memory of their spiritual world.

As Dewey said, “I regard the child's social life as the basis for the concentration or interconnection of all his training or growth. The social life gives him the unconscious unity and context of all his endeavors and his achievements.” The community continues to provide them with experiential resources for physical, cognitive, aesthetic, emotional, and social development. Children perceive the world, develop themselves, and eventually grow into social individuals through the existing “cultural mirror.” The community provides the natural foundation and cultural mirror for children's development and builds a broad platform for children's growth.

The article "Research on the New Ecological Model under the Environment of “Double Reduction” of Children's Community Education Services" was published in 2022. Journal: J Environ Public Health.

## 5. Conclusion

The community is the main place for children's growth and development. The development and utilization of community educational resources can help improve children's emotional experience, enhance children's understanding of nature and society, and promote children to develop good behavior habits and thinking awareness. Therefore, the community should attach importance to the development and utilization of children's educational resources and follow the principle of the subject, fit, and development.

This paper discusses the theoretical basis of the development and utilization of community children's education resources under the dual emission reduction policy, puts forward the corresponding development principles, and analyzes the main strategies to improve the efficiency of social education. First of all, starting from natural resources, guide children to observe nature, understand nature, and apply natural things to innovate and create. Secondly, the community should also strengthen the development and utilization of community space resources to create a good learning environment for children. In addition, the community should increase publicity, mobilize the strength of all sectors of society, and work together for the growth of children.

## Figures and Tables

**Figure 1:** Relevant theoretical basis for the development and utilization of community educational resources.

**Figure 2:** Two important factors in child development.

**Figure 3:** Principles of development and utilization of educational resources for children in the community.

**Figure 4:** Two aspects of the suitability principle.

**Figure 5:** Strategies for the development and utilization of educational resources for children in the community.

**Table 1:** Social education methods.

1	Providing venues and resources for off-campus activities	The youth palaces, youth activity centers, research and practice education bases (camps), museums, and other off-campus activity venues at all levels must adhere to the principle of public welfare and increase the opening hours, especially after 3:30 pm, weekends, winter and summer vacations, etc., are open to primary and secondary school students.

2	Exploring community education services	The community should build a student activity center to provide a place for students to participate in social practice, club activities, and volunteer services after school.

3	Propagating the concept of scientific education	All kinds of news media should actively publicize the concept of scientific education, strive to get rid of utilitarian phenomena, such as “rush-run culture,” do not hype the ranking of test scores and the rate of admission, and create a good atmosphere for social education.

The article "Research on the New Ecological Model under the Environment of “Double Reduction” of Children's Community Education Services" was published in 2022. Journal: J Environ Public Health.

**Table 2:** “Living education” theory.

1	Nature and society are the sources of knowledge, and many human wisdom and creations are condensed in nature and society. Using them as teaching materials for children's education can be more vivid and intuitive while avoiding other forms of distortion and changes. Let children directly feel the correct values

2	Showing educational materials for children in nature and society is richer and can greatly mobilize children's enthusiasm. Children are more willing and accepted to learn knowledge in nature and society, explore the unknown world, and change the rigid and rigid preaching form; the enlightenment to children's souls is more profound and lasting

**Table 3:** Rich types of community public service institutions.

Specialized educational institutions	Kindergartens, schools, libraries, museums, etc.

Specialized medical institutions	Hospitals, clinics, etc.

Specialized commercial institutions	Supermarkets, shopping malls, pharmacies, flower shops, beauty shops, etc.

Special transportation places	Railway stations, bus stations, airports, etc.

Specialized entertainment venues	Opera houses, cinemas, etc.

Specialized occupational places	Police station, fire station, community service center, etc.

## Data Availability

The labeled data set used to support the findings of this study is available from the corresponding author upon request.
